# Wenxin Granules Regulate Endoplasmic Reticulum Stress Unfolded Protein Response and Improve Ventricular Remodeling on Rats with Myocardial Infarction

**DOI:** 10.1155/2021/7375549

**Published:** 2021-11-02

**Authors:** Keke Liu, Meng Lv, Xiaodi Ji, Lixia Lou, Bo Nie, Jiuli Zhao, Aiming Wu, Mingjing Zhao

**Affiliations:** Dongzhimen Hospital Affiliated to Beijing University of Chinese Medicine, Key Laboratory of Chinese Internal Medicine of Ministry of Education and Beijing, Beijing 100700, China

## Abstract

*Background*. Arrhythmia after myocardial infarction is the leading cause of death in clinical heart disease. Increasing studies have shown that the response to endoplasmic reticulum (ER) stress (ERS) caused by myocardial infarction is related to prognosis and the development of arrhythmias. The unfolded protein response (UPR) could serve as an important regulatory signaling pathway following myocardial infarction. The traditional Chinese medicine Wenxin Granules improve arrhythmias following myocardial infarction, which may be related to ERS intervention and the activation of the UPR and apoptosis. We aimed to investigate the involvement of Wenxin Granules in the activation of the UPR and apoptosis following myocardial infarction. Left coronary artery ligation was established as a rat model of myocardial infarction. The rats were randomly divided into the model group, low-dose Wenxin Granule group, high-dose Wenxin Granule group, and metoprolol group. Rats with only wire insertion and no ligature were used as the sham group. Small animal ultrasound systems were used to detect changes in heart structure and function, and the electrical stimulation threshold for ventricular fibrillation was detected. The expression of glucose-regulated protein (GRP)78, activating transcription factor (ATF)6, X-box binding protein (XBP)1, protein kinase–like ER kinase (PERK), phosphorylated (p)-PERK, Bax, Bcl2, C/EBP homologous protein (CHOP), caspase 12, caspase 8, and caspase 3 were detected by western blot, and terminal deoxynucleotidyl transferase dUTP Nick end labeling (TUNEL) was used to determine the cardiomyocyte apoptosis index. Compared with the sham group, rats in the model group displayed immediate ST-segment elevation and pathological *Q* waves after 24 hours. After 2 weeks, the left ventricular (LV) anterior wall thickness (LVAW) became thinner, and the inner diameter (LVID) increased. The end-diastolic LVAW (LVAWd), end-systolic LVAW (LVAWs), ejection fraction (EF), and fractional shortening (FS) were significantly reduced (*P* < 0.01), whereas the LVIDd, LVIDs, diastolic LV volume (LV Vold), and systolic LV volume (LV Vols) significantly increased (*P* < 0.01). The ventricular fibrillation threshold decreased significantly (*P* < 0.01). ERS proteins GRP78, p-PERK, PERK, ATF6, and XBP1 and apoptotic proteins CHOP, Bax, caspase 12, caspase 8, and caspase 3 significantly increased (*P* < 0.01, *P* < 0.05), whereas Bcl-2 expression and the Bcl-2/Bax ratio decreased (*P* < 0.01). Compared with the sham group, LVAWd, LVAWs, FS, and Bcl-2 protein expression were significantly increased in the low-dose Wenxin Granule group (*P* < 0.01, *P* < 0.05), and p-PERK and ATF6 decreased (*P* < 0.01, *P* < 0.05). Compared with the sham group, LVAWd, LVAWs, EF, FS, and the ventricular fibrillation threshold significantly increased in the high-dose Wenxin Granule and metoprolol groups (*P* < 0.01, *P* < 0.05), whereas LVIDs, LV Vols, and ERS proteins were significantly decreased (*P* < 0.01, *P* < 0.05). CHOP, Bax, caspase 12, caspase 8, and caspase 3 protein expression decreased in the Wenxin Granule group (*P* < 0.01, *P* < 0.05), whereas Bcl-2 and the Bcl-2/Bax ratio increased (*P* < 0.01, *P* < 0.05). LVIDd and Bax decreased in the metoprolol group (*P* < 0.01, *P* < 0.05), and the Bcl-2/Bax ratio increased (*P* < 0.05). The cardiomyocyte apoptosis index values for the low- and high-dose Wenxin Granule and metoprolol groups were significantly reduced (*P* < 0.05). This study suggested that the UPR is an essential mechanism underlying pathological injury after myocardial infarction. Wenxin Granule treatment can improve ventricular remodeling and cardiac function and inhibit arrhythmia by preventing excessive ERS from activating the UPR and apoptosis.

## 1. Introduction

Cardiovascular disease is a major cause of morbidity and mortality worldwide, and an urgent need exists for the development of new drug therapies. Growing evidence suggests that traditional Chinese medicine (TCM) can play a preventive or therapeutic role for cardiovascular disease through complex mechanisms, such as inhibiting oxidative stress, mitigating damage due to inflammation, promoting angiogenesis and antiapoptosis activities, and regulating autophagy, the gut microflora, and metabolites [1–4]. TCM has the potential to prevent a variety of cardiovascular diseases, such as hypertension, myocardial infarction, cardiomyopathy, arrhythmias, and cardiac remodeling [5–8].

The endoplasmic reticulum (ER) is the primary site of protein synthesis and transport in eukaryotic cells. When cells are stimulated by internal and external factors, the ER functional balance can change, leading to the activation of the ER stress (ERS) mechanism, resulting in the upregulation of specific ERS genes to restore homeostasis. Under conditions of persistent ERS, cells will initiate apoptosis. The ERS can be divided into the unfolded protein response (UPR), which represents the best-studied ERS mechanism, the ER overload reaction, and the cholesterol regulatory cascade reaction. ERS can activate the UPR through three different signaling pathways, including the ER transmembrane protein kinase inositol-requiring enzyme 1 (IRE1), the double-stranded RNA-dependent protein kinase–like ER kinase (PERK), and activated transcription factor 6 (ATF6). UPR activation regulates protein synthesis, degradation, and secretion to mitigate ERS by altering cellular transcription and translation programs [9–11]. ERS often leads to protein misfolding and UPR activation, and the upregulated expression of UPR components is often used as an ERS indicator. Cells activate different signaling molecules depending on the duration and intensity of ERS, which ultimately determine whether the cell adapts or dies.

ERS has also been found to regulate the inflammatory response and the apoptosis signaling pathway through the UPR, maintaining the dynamic ER balance under normal conditions and adapting to balance induced by external stimuli [10]. Excessive or long-lasting ERS leads to impaired cell function and disease development. The contributions of both intracellular and extracellular stress factors following myocardial infarction lead to the accumulation of misfolded or unfolded proteins in the ER lumen. Early or mild ERS induces the UPR, which promotes correct protein folding to alleviate ERS and plays a protective role. However, long-term or severe ERS can induce apoptosis. ERS is an important pathogenic contributor after myocardial infarction, suggesting that interventions that target UPR-related pathways may be important for the prevention and treatment of myocardial infarction.

The bidirectional function of ERS and the synergistic inflammatory response play complex and critical roles in the occurrence and development of disease. The TCM Wenxin Granules are composed of five drugs: *Codonopsis*, Rhizoma Polygoni, *Panax notoginseng*, Amber, and Gansong. Wenxin Granules replenish qi, activates blood, nourishes yin, removes blood stasis, and restores the pulse, which can be used to reduce the occurrence of arrhythmia [12, 13]. Relevant pharmacological studies have shown that the clinical effects of Wenxin Granules are related to the inhibition of myocardial remodeling and the regulation of cardiac conduction systems [14, 15]. ERS-activated UPR signaling has been identified as the pathological basis damage due to myocardial infarction through effects on myocardial remodeling and ion channel activity [16–18], which are closely related to the occurrence of arrhythmias. However, little work has examined the contributions of the UPR to arrhythmia development. In this study, we used Sprague Dawley rats to construct a rat model of myocardial infarction by ligating the anterior descending branch of the left coronary artery to clarify the induction of ERS and cell damage by myocardial infarction and further investigate the contributions of Wenxin Granules to ERS and cell death induced by myocardial infarction.

## 2. Materials and Methods

### 2.1. Animals

Specific-pathogen-free male Sprague Dawley rats were used at 6 weeks old and weighing 180 ± 20 g. Rats were obtained from the Beijing Weitong Lihua Laboratory Animal Technology Co., Ltd., and were raised in a controlled environment in the animal room of Dongzhimen Hospital of Beijing University of Traditional Chinese Medicine. The animal experiment was approved by the Laboratory Animal Welfare and Ethics Committee of Dongzhimen Hospital, Beijing University of Chinese Medicine (approval number 17-12-01). Experimental animal license number is SCXK (Beijing) 2016–0006.

### 2.2. Medicines

Wenxin Keli (WXKL) Granules were produced by Shandong Buchang Pharmaceutical Co., Ltd. (SFDA approval number Z10950026). The main ingredients and quality control of WXKL were those described previously [19], and the product batch number was 2007005. The medicine consists of *Codonopsis*, *Panax notoginseng*, Amber, Gansong, and *Polygonatum*. Metoprolol tartrate tablets were produced by AstraZeneca Pharmaceutical Co., Ltd. (National Medicine Standard H32025391).

### 2.3. Main Reagents and Instruments

The following reagents and instruments were used: pentobarbital sodium (Beijing Chemical Reagent Company, batch number: C06818794), hematoxylin and eosin (HE) staining solution (Nanjing Jiancheng Technology Co., Ltd., product number: D006), protease phosphatase inhibitor mixture (Beyotime Company, product number: P1045), bicinchoninic acid (BCA) protein concentration determination kit (LABLEAD company, product number: B5000), 4 × sodium dodecyl sulfate (SDS) protein loading buffer (LABLEAD company, product number: G2526-1), glyceraldehyde-3-phosphate dehydrogenase (GAPDH) antibody (Proteintech company, product number: 60004-1-Ig), anti-rabbit secondary antibody, anti-mouse secondary antibody (LABLEAD company, product number: s0101-1, s0100-1), PERK and p-PERK antibodies (CST company, product numbers: 3192s and 3179s, resp.), ATF6 and XBP1 antibodies (Abcam company, product numbers: ab203119 and ab37152, resp.), GRP78, CHOP, Bcl-2, Bax, caspase 3, and caspase 8 antibodies (Proteintech company, product numbers: 11587-1AP, 15204-1-AP, 26591-1-Ap, 60267-1-Ig, 19677-1-AP, and 13423-1-AP, resp.), caspase 12 antibody (Abcam, product number: ab62484), DeadEnd™ terminal deoxynucleotidyl transferase dUTP Nick end labeling (TUNEL) fluorescence detection reagent kit (Promega, product number: G3250), small animal ventilator (Shanghai Alcott Biotechnology Co., Ltd., model number: ALC-V8S), multichannel automatic analysis electrocardiograph (Beijing Futian Electronic Medical Instrument Co., Ltd., model number: FX-7202), biological function experiment signal acquisition system (Chengdu Taimeng Software Co., Ltd., model number: BL-420S), electronic balance (Shanghai Precision Scientific Instrument Co., Ltd., model number: JA1003 N), microplate reader (Thermo Fisher, USA, model number: Varioskan LUX), inverted optical microscope (Olympus, Japan, model number: Olympus BX60), small animal ultrasound system (Visual Sonics, model number: Vevo 2100), electrophoresis tank, and electrorotor tank (Beijing Longfang Technology Co., Ltd., product number: LF-mini3, LF-ZY01).

### 2.4. Model Preparation

A previously published paper [20] was referenced for the establishment of a rat model of myocardial infarction. First, the rats were anesthetized with 1% sodium pentobarbital (0.5 ml/100 g) injected intraperitoneally, fixed in a supine position, and intubated through the larynx and trachea. The third and fourth intercostals of the anterior area were opened laterally. The left anterior descending coronary artery was ligated using a 5/0 surgical suture approximately 2 mm below the pulmonary artery cone and the left atrial appendage. The left ventricular anterior wall (LVAW) became white, and the ST-segment of the electrocardiogram (ECG) became elevated. The chest was closed using sutures, layer by layer. A pathological *Q* wave appeared in the ECG 24 hours after the operation, indicating that the ligation operation was successful. The sham operation group was operated in parallel without ligation. To prevent infection, 40 U penicillin was administered by injection for 3 consecutive days after the operation.

### 2.5. Group Administration

The rats were randomly divided into the sham operation group, the model group, the low-dose Wenxin Granule group, the high-dose Wenxin Granule group, and the metoprolol group. The sham group received the sham operation, and all other groups were subjected to ligation. The Wenxin Granule doses were established according to the “Pharmacological Experiment Methodology” by Xu Shuyun [21], and the human clinical daily dose was converted into an equivalent dose for rats (approximately 6 times the human clinical dose) for the low-dose group, which was doubled for the high-dose group (approximately 12 times the human clinical dose). The metoprolol group received an equivalent dose (approximately 6 times the human clinical dose). Intragastric drug administration was started 24 hours after the operation and was performed once per day for 2 consecutive weeks. The model group and sham operation group were administered an equal volume of deionized water each day.

### 2.6. Small Animal Ultrasound Detection

Two weeks after the operation, 1% sodium pentobarbital was injected intraperitoneally to anesthetize the animals. After skin preparation, the animals were fixed in a dorsal position to perform ECG. The MS201 probe was placed on the left chest of the rat to obtain a satisfactory two-dimensional image of the long-axis of the left ventricle (LV). The probe was rotated 90° clockwise to obtain the short-axis view at the level of the papillary muscle. The short-axis LVAW end-diastolic thickness (LVAWd), LVAW end-systolic thickness (LVAWs), left ventricular inner diameter end-diastolic thickness (LVIDd), left ventricular end-systolic thickness (LVIDs), posterior wall end-diastolic thickness (LVPWd), posterior wall end-systolic thickness (LVPWs), left ventricular ejection fraction (EF), fractional shortening (FS), diastolic left ventricular volume (LV Vold), and systolic left ventricular volume (LV Vols) were measured 5 times for each animal, and the average was used as a representative value.

### 2.7. The Ventricular Electrical Stimulation Fibrillation Threshold

First, a cut was made between ribs 4 and 5 of the rat chest, and two pairs of tweezers were used to bluntly separate the muscles and ribs. After fully exposing the heart, the apex of the heart was connected to the positive pole of the stimulating electrode, and the negative pole was connected to the bottom of the heart, approximately 3 mm away from the positive pole. BL-420 software was used in stimulation mode, using the following parameters: (a) mode: coarse voltage; (b) delay: 5 ms; (c) frequency: 30 Hz; (d) method: string stimulation; (e) wave width: 5 ms; (f) intensity: 1 V; and (g) string length: 10 stimulation waves. Program control information was set according to the following parameters: (a) type: automatic amplitude direction increase; (b) increment: 1 V; (c) main period: 10 seconds; and (d): number of stops: 20. According to the ECG results, the voltage of ventricular fibrillation first appeared as a ventricular threshold.

### 2.8. Western Blot

The radioimmunoprecipitation assay (RIPA) protein lysis method was used to extract the total protein from the tissue, and the BCA method was used to determine the protein concentration. All protein samples were adjusted to the same concentration according to the measurement results and stored at −20°C. Western blot assays were performed within 2 weeks of protein lysis. SDS-polyacrylamide gel electrophoresis (PAGE) was used to separate the proteins, followed by a wet transfer to a nitrocellulose membrane, which was blocked in 5% skim milk at room temperature with shaking for 1 h. Membranes were incubated with preconfigured primary antibodies overnight at 4°C. The next day, after washing the membrane with Tris-buffered saline containing Tween 20 (TBST), the corresponding secondary antibody was added and incubated for 1 h at room temperature. After washing with TBST, the protein band was visualized using enhanced chemiluminescence (ECL). ImageJ was used to analyze the bands using GAPDH as the internal reference.

### 2.9. TUNEL Method to Determine the Cell Apoptosis Index

TUNEL staining was performed according to the kit instructions. Sections were fully deparaffinized, hydrated, and fixed in 4% paraformaldehyde for 15 min. Sections were washed with phosphate-buffered saline (PBS) and incubated with 20 *μ*g/ml proteinase K at room temperature for 10 min. The balance solution was equilibrated at room temperature for 10 min, and the reaction solution was prepared on ice, followed by incubation at 37°C for 60 min. The stop solution was added for 15 min, and sections were washed with PBS solution to remove unincorporated fluorescein-12-dUTP. A drop of anti-fluorescence attenuation sealing liquid containing 4′,6-diamidino-2-phenylindole (DAPI) was added to the myocardial tissue, which was sealed with cover glass. Image acquisition was performed immediately under a fluorescence microscope (A1, ZEISS, Germany), using a standard fluorescein filter to observe green fluorescence at 520 nm, which visualized apoptotic nuclei; intact blue nuclei were visualized at 460 nm. ImageJ software was used to count the numbers of apoptotic cell nuclei and normal cell nuclei to calculate the apoptosis index.

### 2.10. Statistical Analysis

SPSS 23.0 software was used for all statistical analyses. Data conforming to the normal distribution are expressed as the mean ± standard deviation and assessed by one-way analysis of variance (ANOVA). Comparisons between groups were performed using the least significant difference (LSD) method. The Kruskal–Wallis rank-sum test was used for comparisons between groups that did not conform to the normal distribution. *P* < 0.05 was considered significant.

## 3. Results

### 3.1. ECG Results of Rats in the Sham Operation and Model Groups

Compared with the sham operation group, the rats in the model group presented with ST-segment elevation immediately after the operation, and a pathological *Q* wave appeared 24 hours after the operation (Figure 1(a)).

### 3.2. Comparison of Gross Cardiac Results

Compared with the sham operation group, the model group had larger hearts, and the LVAW became thinner, whereas each treatment group showed improvements relative to the model group, to some extent (Figure 1(b)).

### 3.3. HE Staining

The myocardial cells derived from the sham operation group presented with normal morphology, with the myocardial fibers arranged neatly and stained uniformly, and the nuclear morphology was normal. Compared with the sham operation group, the model group presented with a large necrotic area in the myocardial tissue and pyknosis of the nucleus. The remaining myocardium presented with a disordered arrangement. Compared with the model group, the treatment groups showed reductions in the observed pathological changes (Figure 1(c)).

### 3.4. Comparison of Ultrasound Detection Results in Rats

Compared with the sham operation group, the LVAW in the model group became thinner, and the LVID increased 2 weeks after the operation (Figure 2(a)). The LVAWd and LVAWs were significantly reduced (*P* < 0.01), the LVIDd and LVIDs were significantly increased (*P* < 0.01), the EF and FS were significantly reduced (*P* < 0.01), and the LV Vold and LV Vols were significantly increased (*P* < 0.01). Compared with the sham operation group, the low-dose Wenxin Granule group showed a significant increase in LVAWd, LVAWs, and FS (*P* < 0.01, *P* < 0.05). The high-dose Wenxin Granule group and the metoprolol group presented with significantly increased values for LVAWd, LVAWs, EF, and FS (*P* < 0.01), whereas LVIDs and LV Vols were significantly decreased (*P* < 0.01, *P* < 0.05). In addition, the metoprolol group showed a significantly decreased LVIDd (*P* < 0.01) (Figure 2(b)).

### 3.5. Comparison of Ventricular Fibrillation Threshold

Compared with the sham operation group, the ventricular fibrillation threshold of the model group was significantly lower (*P* < 0.01). Compared with the model group, the high-dose Wenxin Granule group and the metoprolol group had significantly increased ventricular fibrillation thresholds (*P* < 0.01, *P* < 0.05). The low-dose Wenxin Granule group increased the ventricular fibrillation threshold, but not significantly (Figures 3(a) and 3(b)).

### 3.6. Influence of Wenxin Granules on the Expression of Key UPR Protein GRP78 under ERS Conditions

Compared with the sham operation group, the expression of GRP78 in the model group was significantly increased (*P* < 0.01), whereas the expression of GRP78 in each treatment group was significantly decreased compared with that in the model group (*P* < 0.01) (Figures 4(a) and (b)).

### 3.7. Comparison of the Expression of UPR Cascade-Related Proteins

Compared with the sham operation group, the expression levels of ERS proteins GRP78, p-PERK, PERK, ATF6, and XBP1 in the model group were significantly increased (*P* < 0.01). Compared with the model group, expression levels of p-PERK and ATF6 in the low-dose Wenxin Granule group were significantly reduced (*P* < 0.01, *P* < 0.05). Although the other proteins displayed a decreasing trend, they did not reach significance. The expression levels of the ERS pathway proteins were all significantly decreased in the high-dose Wenxin Granule and metoprolol groups compared with the model group (*P* < 0.01, *P* < 0.05) (Figures 5(a) and 5(b)).

### 3.8. Comparison of Apoptosis-Related Proteins

Compared with the sham operation group, the expression levels of apoptotic proteins, including CHOP, Bax, caspase 12, caspase 8, and caspase 3, were significantly increased in the model group (*P* < 0.01, *P* < 0.05), whereas the expression levels of Bcl-2 and the ratio of Bcl-2/Bax were significantly decreased (*P* < 0.01). Compared with the model group, the expression level of Bcl-2 protein in the low-dose Wenxin Granule group increased (*P* < 0.05), whereas the expression levels of other apoptotic proteins were not significantly different. The protein expression levels of CHOP, Bax, caspase 12, caspase 8, and caspase 3 in the high-dose Wenxin Granule group were significantly decreased compared with those in the model group (*P* < 0.01, *P* < 0.05), whereas the protein expression level of Bcl-2 and the Bcl-2/Bax ratio were significantly increased (*P* < 0.01, *P* < 0.05). The expression level of Bax protein in the metoprolol group was significantly decreased compared with that in the model group (*P* < 0.05), whereas the Bcl-2/Bax ratio was significantly increased (*P* < 0.05) (Figures 6(a)–6(c)).

### 3.9. The Apoptosis Index of Myocardial Cells by TUNEL Staining

Compared with the sham operation group, the apoptosis index of cardiomyocytes from the model group was significantly increased (*P* < 0.01). Compared with the model group, the apoptosis index values for cardiomyocytes in the low- and high-dose Wenxin Granule groups and the metoprolol group were significantly decreased (*P* < 0.05) (Figures 7(a) and 7(b)).

## 4. Discussion

In this study, the myocardial infarction rat model was established by ligating the anterior descending branch of the left coronary artery in Sprague Dawley rats. Both gross heart observations and HE staining showed that the induction of myocardial infarction caused serious histopathological damage, which was reduced by treatment with Wenxin Granules, indicating that Wenxin Granules could play a potentially protective role (Figure 1).

The cardioprotective effects of Wenxin Granules are related to improving ventricular reconstruction, improving heart function, and inhibiting the occurrence of arrhythmia. Ventricular remodeling occurs following myocardial infarction, including increased LV Vol and changes in the shape and thickness of the infarcted myocardium, which influences the contractile and electrical activity of the ventricle. Cardiac remodeling is the most important and representative change that occurs following myocardial infarction, resulting in the further deterioration of cardiac function. The results showed that Wenxin Granule treatment could improve cardiac function in a dose-dependent manner, increasing the thickness of the LVAW, reducing the LVID, improving the cardiac EF, and inducing FS (Figure 2). Studies have confirmed that the cardioprotective effects of Wenxin Granules are related to the repair of ischemic and necrotic myocardial tissue after myocardial infarction, improving cardiac function, and reducing the occurrence of arrhythmia [12, 13, 15, 19]. The ventricular fibrillation threshold was measured by electrical stimulation, which showed that Wenxin Granule treatment increased the ventricular fibrillation threshold, reducing the occurrence of arrhythmias (Figure 3).

The ERS response is a primary pathological mechanism associated with myocardial infarction [22–24], and Wenxin Granules may play a protective role by reducing the activation of the UPR under ERS conditions. The ERS-initiated UPR exerts biological effects through three pathways: IRE1, PERK, and ATF6. Under physiological conditions, GRP78 binds to PERK, IRE1, or ATF6 to form a stable and inactive complex, limiting the transmission of the corresponding downstream signals. When the UPR is initiated, GRP78 disassociates from these three proteins and binds to unfolded or misfolded proteins, activating downstream cascade reactions and causing changes in the expression patterns of related proteins, such as GRP78, PERK, ATF6, and XBP1 [11, 25, 26]. Myocardial infarction induces ERS by interfering with the formation of oxygen-dependent disulfide bonds after translation, disrupts protein folding and isomerization after translation, and affects the formation of oxygen-dependent disulfide bonds. In addition, the lack of glucose or glutamine caused by ischemia can interrupt the hexosamine biosynthetic pathway, which requires these two nutrients to produce uridine diphosphate-N-acetylglucosamine (UDP-GlcNAc), a necessary factor in N-chain glycosylation and protein folding in the ER [27]. Myocardial infarction causes the abnormal activation of the UPR and the significantly increased expression of ERS proteins, including GRP78, PERK, ATF6, XBP1, and p-PERK, indicating that myocardial infarction triggered the excessive activation of the ERS pathway (Figure 5). Continuous and severe ERS eventually activates the apoptotic pathway, aggravating pathological damage in the heart tissue. Apoptosis induced by ERS requires specific signaling pathways, including the CHOP pathway, the Bcl-2 family, and caspase 12 activation.

Excessive UPR leads to the activation of apoptosis-related genes. Activated IRE1, ATF6, and PERK can all induce the generation of CHOP, which promotes the release of mitochondrial cytoplasmic C, the formation of apoptotic bodies, and the activation of the caspase cascade to induce apoptosis by upregulating the expression of the proapoptotic protein Bax and downregulating the expression of Bcl-2 [28, 29]. In this experiment, the expression levels of apoptotic proteins CHOP and Bax in the model group significantly increased (*P* < 0.01) compared with the sham group, whereas the expression level of Bcl-2 and the Bcl-2/Bax ratio significantly decreased (*P* < 0.01, Figure 6). Excessive UPR activation results in the activation of apoptosis-related genes, and eventually, the activation of the caspase cascade leads to apoptosis [30]. Two main caspase pathways have been identified. One pathway is mediated by the death domain, in which the death signal molecule binds to its receptor to induce caspase 8 to autocatalyze into a protease with hydrolase activity; caspase 8 can then hydrolyze the downstream caspases 3, 6, and 7, which act on the substrate to degrade it, leading to cell apoptosis [28]. The other pathway is mediated by the mitochondrial cytochrome C activation of caspase 9, which, in turn, activates caspase 3 [31]. In addition, caspase 12 activation serves as a marker of the ERS-specific apoptotic pathway [28, 32]. The expression levels of the apoptotic proteins caspase 12, caspase 8, and caspase 3 were significantly increased in the model group compared with those in the sham group (*P* < 0.01, *P* < 0.05; Figure 6). Wenxin Granules played a protective role by downregulating the expression of related proteins, inhibiting ERS-mediated apoptosis. The TUNEL assay also showed that Wenxin Granules could significantly reduce apoptosis in cardiomyocytes (*P* < 0.05, Figure 7).

In the last decade, great progress has been made in the field of modern medicine, but many treatment methods have encountered technological difficulties or come at great cost. The integration of modern medicine with TCM is likely to result in beneficial effects for the treatment of myocardial infarction. In summary, this study revealed that Wenxin Granules induce beneficial effects through the regulation of ERS-mediated UPR activation, which can guide further research regarding the molecular regulatory mechanisms that can be targeted for the prevention and treatment of myocardial infarction. Treatment with Wenxin Granules was able to improve ventricular remodeling and cardiac function and inhibit arrhythmia by alleviating the pathological damage caused by myocardial infarction, the inhibition of excessive ERS-mediated UPR activation, and the reduction of myocardial cell apoptosis.

## 5. Conclusion

Wenxin Granule treatment can improve ventricular remodeling and cardiac functions and inhibit arrhythmia by preventing excessive ERS-mediated activation of the UPR and apoptosis.

## Figures and Tables

**Figure 1:** ECG recordings from rats and the pathological changes in the left ventricular myocardium. (a) ECG results from rats in the sham operation group and the model group. (b) Comparison of gross cardiac results. (c) Hematoxylin and eosin staining results from rats in each group 2 weeks after surgery (400×). Pre: before surgery; Im; immediately after surgery; A: sham operation group; B: model group; C: low-dose Wenxin Granule group; D: high-dose Wenxin Granule group; E: metoprolol group.

**Figure 2:** Comparison of cardiac structure and function in rats (*n* = 8). (a) Comparison of ultrasound detection results of rats from each group. (b) Comparisons of heart functions and left ventricular thickness in rats. The data are expressed as the mean ± SD. A: sham operation group; B: model group; C: low-dose Wenxin Granule group; D: high-dose Wenxin Granule group; E: metoprolol group. ^*∗*^*P* < 0.05, ^∗∗^*P* < 0.01 compared with the sham operation group, ^#^*P* < 0.05, ^##^*P* < 0.01 compared with the model group. LVAWd: short-axis left ventricular atrial wall end-diastolic thickness; LVAWs: short-axis left ventricular atrial wall end-systolic thickness; LVIDd: left ventricular inner diameter end-diastolic thickness; LVIDs: left ventricular end-systolic thickness; LVPWd: posterior wall end-diastolic thickness; LVPWs: posterior wall end-systolic thickness LV Vold: diastolic left ventricular volume; LV Vols: systolic left ventricular volume.

**Figure 3:** Comparison of ventricular fibrillation thresholds (*n* = 7). To confirm the benefits of Wenxin Granule treatment for mitigating potentially lethal arrhythmias following myocardial infarction (MI), programmatic electrophysiological stimulation was performed 2 weeks after MI *in vivo*. (a) The compressed waveform of the epicardial electrogram recording and the expanded waveform. (b) Comparison of ventricular fibrillation threshold values, expressed as the mean ± SD. A: sham operation group; B: model group; C: low-dose Wenxin Granule group; D: high-dose Wenxin Granule group; E: metoprolol group. , ^*∗*^*P* < 0.05, ^∗∗^*P* < 0.01 compared with the sham operation group, ^#^*P* < 0.05, ^##^*P* < 0.01 compared with the model group.

**Figure 4:** Comparison of the expression of a key unfolded protein response (UPR) protein, glucose-regulated protein 78 (GRP78). (a) The immunohistochemical expression of the key UPR protein GRP78 (200×). (b) Comparison of GRP78 values expressed as the mean ± SD (*n* = 7). A: sham operation group; B: model group; C: low-dose Wenxin Granule group; D: high-dose Wenxin Granule group; E: metoprolol group. ^*∗*^*P* < 0.05, ^∗∗^*P* < 0.01 compared with the sham operation group, ^#^*P* < 0.05, ^##^*P* < 0.01 compared with the model group.

**Figure 5:** Comparison of unfolded protein response- (UPR-) related protein expression. (a) Comparisons of UPR-related protein expression levels. (b) Comparison of UPR-related protein values expressed as the mean ± SD (*n* = 6). A: sham operation group; B: model group; C: low-dose Wenxin Granule group; D: high-dose Wenxin Granule group; E: metoprolol group. ^*∗*^*P* < 0.05, ^∗∗^*P* < 0.01 compared with the sham operation group, ^#^*P* < 0.05, ^##^*P* < 0.01 compared with the model group. GRP78: glucose-regulated protein 78; p-PERK: phosphorylated protein kinase RNA-like endoplasmic reticulum kinase; ATF6: activated transcription factor 6; XBP1: X-box binding protein 1.

**Figure 6:** Comparison of apoptosis-related proteins (*n* = 6). (a) Comparison of apoptosis-related proteins. (b) Comparison of apoptosis-related protein values, expressed as the mean ± SD (*n* = 6). A: sham operation group; B: model group; C: low-dose Wenxin Granule group; D: high-dose Wenxin Granule group; E: metoprolol group. ^*∗*^*P* < 0.05, ^∗∗^*P* < 0.01 compared with the sham operation group, ^#^*P* < 0.05, ^##^*P* < 0.01 compared with the model group (c).

**Figure 7:** Comparison of myocardial cell apoptosis detected by terminal deoxynucleotidyl transferase dUTP Nick end labeling (TUNEL). (a) Comparison of myocardial cell apoptosis (400×). (b) Comparison of myocardial cell apoptosis values expressed as the mean ± SD (*n* = 8). A: sham operation group; B: model group; C: low-dose Wenxin Granule group; D: high-dose Wenxin Granule group; E: metoprolol group. ^*∗*^*P* < 0.05, ^∗∗^*P* < 0.01 compared with the sham operation group, ^#^*P* < 0.05, ^##^*P* < 0.01 compared with the model group.

## Data Availability

The data used to support the findings of this study are available from the corresponding author upon request.
